The article "Effect of Eriodictyol on Retinoblastoma via the PI3K/Akt Pathway" was retracted in 2023. Reasons: signs of a paper mill; suspected computer-generated content; unreliable results or conclusions; lack of ethics approval or compliance.

# Effect of Eriodictyol on Retinoblastoma via the PI3K/Akt Pathway

**DOI:** 10.1155/2021/6091585

**Published:** 2021-11-11

**Authors:** Shu Wen, Meng Hu, Yan Xiong

**Affiliations:** Department of Ophthalmology, Jingmen No. 1 People's Hospital, Xiangshan Road, Jingmen, Hubei, China

## Abstract

Retinoblastoma (RB) is one of the most common intraocular malignancies in children, which causes vision loss and even threatens life. Eriodictyol is a natural flavonoid with strong anticancer activity. Some studies have shown that eriodictyol exerts anticancer effects in glioma, colon cancer, and lung cancer; however, no studies have reported the anticancer effects of eriodictyol on RB. Therefore, the aim of this study was to investigate the anticancer activity of eriodictyol against the RB Y79 cell line and its potential mechanism of action. Interestingly, we found that eriodictyol inhibited the proliferation, migration, and invasion of Y79 cells in a dose-dependent manner and decreased the expression of MMP-2 and MMP-9 proteins in the cells. In addition, eriodictyol-induced apoptosis in Y79 cells was assessed by flow cytometry and immunoblotting. Here, our study revealed that eriodictyol dose dependently inhibited the activation of the PI3K/Akt signaling pathway. Notably, the effect of eriodictyol on RB apoptosis was reversed by a PI3K agonist 740 Y-P. In conclusion, our study shows that eriodictyol effectively inhibits proliferation, migration, and invasion and induces apoptosis in RB cell lines, which may be the result of blocking the PI3K/Akt signaling pathway. Thus, eriodictyol may provide a new theoretical basis for exploring targeted antitumor natural therapies.

## 1. Introduction

Retinoblastoma (Rb) is one of the most common intraocular malignancies in children due to mutations in the oncogene RB1, which accounts for approximately 4% of all pediatric malignancies [1, 2]. Currently, protection of the ocular body, improvement of visual acuity, and prevention of metastatic disease are the main treatments for RB. Chemotherapy (intravenous, intra-arterial, and intraocular), local therapies (cryotherapy and transpupillary thermotherapy), radiotherapy (external radiation radiotherapy and plaque radiotherapy), and global extraction are commonly used in clinical practice [3]. Although numerous treatment options can improve the survival rate of RB patients, the efficacy is often affected by the duration of the disease, developmental limitations of the economic situation in different countries, drug resistance, and drug side effects. Therefore, exploring new drug targets and improving efficacy are new strategies for the treatment of RB at present.

Eriodictyol is a natural dihydroflavonoid widely found in vegetables, fruits, and herbs [4]. In North America, eriodictyol-rich plants are often used by Indians as medicine for diseases such as rheumatism, asthma, and allergic rhinitis. In recent years, as the research on eriodictyol has intensified, more and more researchers have found that it has various pharmacological activities such as antioxidant, anti-inflammatory, metabolic modulation, and neuroprotection [5–8]. However, recent studies have found that *Saccharomyces cerevisiae* can inhibit glioma cell proliferation and metastasis and induce apoptosis through the PI3K/Akt signaling pathway [9] in addition to its strong anticancer activity in lung, nasopharyngeal, and colon cancers [10–14].

The article "Effect of Eriodictyol on Retinoblastoma via the PI3K/Akt Pathway" was retracted in 2023. Reasons: signs of a paper mill; suspected computer-generated content; unreliable results or conclusions; lack of ethics approval or compliance.

The PI3K/Akt signaling pathway is a classical signaling pathway involved in the regulation of cell survival, proliferation, apoptosis, and angiogenesis [15]. Current studies have shown that abnormal activation of the PI3K/Akt signaling pathway is closely related to the development of malignant tumors, and it plays an important role in tumor cell proliferation, migration, and degradation of the extracellular matrix [16]. When stimulated by upstream signals such as growth factors, PI3K activates Akt, which further activates various protein molecules downstream such as caspase-3, MMP-2, and MMP-9 to regulate tumor cell proliferation, invasion, and metastasis, apoptosis, angiogenesis, and glycolytic metabolism [17, 18]. Notably, tumor therapeutic regimens targeting PI3K-mediated signaling pathways are currently a hot research topic at home and abroad, and inhibitors and activators targeting individual signaling molecules in the PI3K/Akt pathway are increasingly used in clinical trials [19, 20].

Currently, some studies have reported that the PI3K/Akt pathway plays an important role in RB [21–23]; however, the anticancer effect of eriodictyol on RB has not been reported. The purpose of this study was to investigate the antitumor effect of eriodictyol on the retinoblastoma Y79 cell line and its potential mechanism of action and to provide a new basis for tumor therapy with the PI3K-Akt signaling pathway as a key molecular target.

## 2. Materials and Methods

### 2.1. Materials

Retinoblastoma Y79 cell line was purchased from American Culture Collection (ATCC, HTB-169, Manassas, VA, USA). Eriodictyol (purity ≥98%) was purchased from Dalian Meilun Biotechnology Co. Rabbit anti-human, MMP-2, and MMP-9 antibodies were purchased from Santa Cruz (Dallas, TX, USA). Anti-*β*-actin, Akt, P-Akt, PI3K, caspase-3, MMP-2, and MMP-9 antibodies were purchased from Abcam (Shanghai, China). Cell culture medium (RPMI-1640) and fetal bovine serum were purchased from Gibco, Thermo Fisher Scientific (Grand Island, NY, USA). All other reagents were purchased from Sangon Biotech (Shanghai, China).

The article "Effect of Eriodictyol on Retinoblastoma via the PI3K/Akt Pathway" was retracted in 2023. Reasons: signs of a paper mill; suspected computer-generated content; unreliable results or conclusions; lack of ethics approval or compliance.

### 2.2. Cell Culture and Eriodictyol Treatment

Retinoblastoma (RB) tumor cell line Y79 was purchased from the American Typical Culture Collection (ATCC, Manassas, VA). All cells were cultured in the DMEM containing 10% fetal bovine serum (FBS, Biological Industries, Kibbutz Beit-HaEmek, Israel) and 1% penicillin/streptomycin at 5% CO_2_ and 37°C.

### 2.3. CCK-8 Method to Detect the Effect of Different Concentrations of Eriodictyol on the Proliferation of Y79 Cells

Retinoblastoma Y79 cells were inoculated into 96-well plates at a density of 1 × 10^4^ cells per well, incubated overnight in a CO_2_ incubator, and then treated with a complete medium containing different concentrations of eriodictyol (0 *μ*M, 25 *μ*M, 50 *μ*M, and 100 *μ*M) for 48 h. After discarding the medium, the cells were washed with PBS 2-3 times. Then, 100 *μ*L of the medium containing 10% CCK-8 was added to each well and incubated in a CO_2_ incubator for 2 h. Finally, the OD at 450 nm was measured using an enzyme marker, and cell viability was calculated.

### 2.4. Effect of Eriodictyol on the Migration of Retinoblastoma Cells

Cell migration was assessed using the transwell method. Y79-RB cells were cultured with different concentrations of eriodictyol, and cells were digested with trypsin and suspended in the medium at a density of 1 × 10^5^ cells/well. Y79-RB cells were spread on the top wells of transwell plates (200 *μ*L/well) coated with Matrigel on top. Bottom wells were added with 500 *μ*L of the cell culture medium, and after 24 hours of incubation at 37°C, unmigrated cells were removed from the top side of each chamber with a cotton swab. The cells were fixed with 4% paraformaldehyde for 30 min at room temperature and then stained with 0.5% crystal violet for 15 min. Images were taken using a Leica DMI3000B microscope, and migrating cells were counted at 100x magnification.

### 2.5. Effect of Eriodictyol on Retinoblastoma Cell Invasion

The invasive ability of cells was assayed using Matrigel-coated transwell chambers. After preparing a mixed matrix gel solution according to the ratio of Matrigel : DMEM = 1 : 8, 60 *μ*L mixed solution was added to each of the upper chambers of the transwell. Cells in the medium without FBS (5 × 10^4^) were incubated for 4 h at 5% CO_2_ and 37°C. Cells (5 × 10^4^) were inoculated into the top chamber of 8 *μ*m-well transwell inserts (Corning) in 24-well plates. The FBS-containing medium was added to the bottom chamber. After 24 h incubation with eriodictyol, the small chambers were fixed with 4% paraformaldehyde and stained with 0.1% crystalline violet and wiped from the top of the upper chamber for cells that had not been invaded. Images were taken using a Leica DMI3000B microscope, and the results were counted.

The article "Effect of Eriodictyol on Retinoblastoma via the PI3K/Akt Pathway" was retracted in 2023. Reasons: signs of a paper mill; suspected computer-generated content; unreliable results or conclusions; lack of ethics approval or compliance.

### 2.6. Effect of Eriodictyol on Apoptosis of Retinoblastoma Cells

Retinoblastoma Y79 cell line was collected at a cell count of approximately 5 × 10^6^ cells/mL in a centrifuge tube, centrifuged at 1000 r/min for 5 min, discarded, washed once with 3 mL PBS, centrifuged and discarded, and fixed with ice-precooled 70% ethanol at 4°C for 2 hours. Centrifuge and discard the fixative, and resuspend 3 ml of PBS for 5 min. 400-mesh sieve filter once, centrifuge at 500–1000 r/min for 5 min, discard PBS, stain with 1 mL of PI staining solution, and incubate at 4°C for 30 min protected from light. PI fluorescence is excited with the argon ion, the laser light wave wavelength is 488 nm, and the wavelength of the emitted light wave is greater than 630 nm. The histogram of the fluorescence intensity of PI was analyzed by generating red fluorescence.

### 2.7. Western Blot for the Effect of Eriodictyol on the Expression of Y79 Cell-Associated Proteins

Retinoblastoma Y79 cell line was inoculated at a density of 2.5 × 10^5^ cells/ml in 24-well plates at 1 mL per well. Control, dosing, and agonist groups were set up, and after the cells were walled, different concentrations of eriodictyol were given to the dosing group, equal amounts of the complete medium were given to the control group, and PI3K agonist 740YP was added to the agonist group at the same time as the dosing. The cell lysates of each group were extracted for total protein, and the protein concentration was determined by the BCA kit. The denatured protein samples were separated by 10% SDS-PAGE for electrophoresis, and the fully separated proteins in SDS-PAGE were transferred to activated PVDF (polyvinylidene fluoride) membranes, which were closed with 5% skimmed milk powder for 1 h at room temperature and washed three times with TBST. The membranes were incubated overnight at 4°C with primary antibodies for MMP-2, MMP-9, caspase-3, P-PI3K, PI3K, P-Akt, Akt, and *β*-actin, respectively, and washed with TBST the next day, followed by the addition of secondary antibodies labeled with horseradish peroxidase and incubation on a shaker for 2 h. After washing the membranes three times with TBST, the membranes were incubated for 2 h. ECL chemiluminescence reagent was added and developed with a Bio-Rad gel imager. The target protein bands were analyzed semiquantitatively using Image Lab software with *β*-actin as the internal reference.

### 2.8. Statistical Analysis

The data were statistically analyzed using GraphPad Prism 2.0 software, and all results were expressed as mean ± standard deviation (*X* ± SD). *t*-test was used for comparison between two groups of data, and one-way analysis of variance (ANOVA) was used for multiple groups of data. SPSS version 20.0 software (SPSS Inc., Chicago, IL) was used for all statistical analyses. *P* < 0.05 was considered as a statistically significant difference.

The article "Effect of Eriodictyol on Retinoblastoma via the PI3K/Akt Pathway" was retracted in 2023. Reasons: signs of a paper mill; suspected computer-generated content; unreliable results or conclusions; lack of ethics approval or compliance.

## 3. Results and Analysis

### 3.1. Eriodictyol Inhibits the Proliferation of Retinoblastoma Cells

As shown in Figure 1(a), CCK-8 results showed that eriodictyol treatment at 25 *μ*M, 50 *μ*M, and 100 *μ*M significantly inhibited the survival of retinoblastoma Y79 cells for 48 h compared with the control group, and the inhibitory effect on cell proliferation was dose dependent. As shown in Figure 1(b), western blot results showed that compared with the control group, the eriodictyol treatment significantly reduced the expression level of PCNA protein in retinoblastoma Y79 cells, and the inhibitory effect on PCNA protein was dose dependent.

### 3.2. Eriodictyol Inhibits the Migration of Retinoblastoma Cells

As shown in Figure 2, transwell migration results showed that treatment with 25 *μ*M, 50 *μ*M, and 100 *μ*M eriodictyol for 48 h significantly inhibited the ability of retinoblastoma Y79 cells to migrate compared with the control group, and the ability to inhibit cell migration was somewhat dose dependent.

### 3.3. Inhibition of Retinoblastoma Cell Invasion by Eriodictyol

As shown in Figure 3(a), transwell invasion results showed that eriodictyol treatment at 25 *μ*M, 50 *μ*M, and 100 *μ*M significantly inhibited the invasive ability of retinoblastoma Y79 cells for 48 h compared with the control group, and the inhibition of cell invasion was dose dependent. As shown in Figure 3(b), western blot results showed that eriodictyol pretreatment for 48 h significantly reduced the expression levels of MMP-2 and MMP-9 proteins in retinoblastoma Y79 cells, and the inhibition of MMP-2 and MMP-9 proteins had a dose-dependent effect.

### 3.4. Eriodictyol Induces Apoptosis in Retinoblastoma Cells

As shown in Figures 4(a) and 4(b), flow cytometry results showed that eriodictyol at 25 *μ*M, 50 *μ*M, and 100 *μ*M significantly promoted apoptosis of retinoblastoma Y79 cells compared with the control group, and the ability to promote apoptosis was dose dependent. As shown in Figure 4(c), the western blot results showed that eriodictyol treatment significantly increased the expression level of cleaved caspase-3 protein in retinoblastoma Y79 cells, and the promotion of cleaved caspase-3 protein had a dose-dependent effect.

### 3.5. Eriodictyol Inhibits the PI3K/Akt Pathway in Retinoblastoma

As shown in Figure 5(a), western blot results showed that eriodictyol significantly reduced the expression levels of PI3K, Akt, P-PI3K, and P-Akt in retinoblastoma Y79 cells in a dose-dependent way. At the same time, as shown in Figure 5(b), western blot results showed that eriodictyol significantly reduced the expression levels of P-PI3K/PI3K and P-Akt/Akt protein expression ratio in retinoblastoma Y79 cells in a dose-dependent way. It suggests that eriodictyol can inhibit the activation of the PI3K/Akt pathway in retinoblastoma.

The article "Effect of Eriodictyol on Retinoblastoma via the PI3K/Akt Pathway" was retracted in 2023. Reasons: signs of a paper mill; suspected computer-generated content; unreliable results or conclusions; lack of ethics approval or compliance.

### 3.6. Eriodictyol Exerts Antitumor Effects in Retinoblastoma through Inhibition of the PI3K/Akt Pathway

As shown in Figure 6(a), western blot results showed the expression levels of P-PI3K, PI3K, and P-Akt proteins in different groups, 100 *μ*M of eriodictyol significantly decreased the expression levels of cellular P-PI3K/PI3K proteins, and the expression levels of P-PI3K/Akt proteins increased significantly after administration of the PI3K agonist 740 Y-P compared with the administered group.

As shown in Figure 6(b), CCK-8 results showed that 100 *μ*M of eriodictyol significantly inhibited the proliferation of retinoblastoma Y79 cells, and the inhibitory effect of eriodictyol on cell proliferation was reversed after administration of the PI3K agonist 740 Y-P concomitantly.

As shown in Figures 6(c) and 6(d), the transwell migration and transwell invasion results showed that 100 *μ*M of eriodictyol significantly inhibited the ability of retinoblastoma cells to migrate and invade, and after administration of the PI3K agonist 740 Y-P, the effect of eriodictyol on cell migration and invasive ability was reversed.

As shown in Figure 6(e), flow cytometry results showed that 100 *μ*M of eriodictyol significantly promoted apoptosis in retinoblastoma Y79 cells, and administration of the PI3K agonist 740 Y-P significantly reduced the degree of apoptosis.

In this study, we first evaluated the anticancer (cell proliferation, migration, invasion, and apoptosis) effects of eriodictyol on RB.

We treated the RB Y79 cell line with different concentrations of eriodictyol (0 *μ*M, 25 *μ*M, 50 *μ*M, and 100 *μ*M). We first assessed the proliferative effect of eriodictyol on RB cells by detecting CCK-8 and PCNA protein expression levels. Based on the results of previous experiments we selected 48 h as the optimal time for cell proliferation, migration, and invasion of the Y79 cell line in the culture. Among them, the PCNA protein expression level can be used as an assessment index to determine cell proliferation, tumor malignancy, and prognosis [24]. The results of our study showed that eriodictyol dose dependently decreased the survival rate and PCNA protein expression level of RB cells. These findings suggest that eriodictyol can inhibit cell proliferation of RB in a dose-dependent manner.

The article "Effect of Eriodictyol on Retinoblastoma via the PI3K/Akt Pathway" was retracted in 2023. Reasons: signs of a paper mill; suspected computer-generated content; unreliable results or conclusions; lack of ethics approval or compliance.

Current RB therapies mainly block tumor cell division and tumor growth, but there is a lack of specific therapies to block RB metastasis. Therefore, effective inhibition of RB cell invasion and migration is important to improve the prognosis of RB patients. Currently, matrix metalloproteinases (MMPs) play an important role in physiology and pathology by promoting cell proliferation, angiogenesis, invasion, and reduction of migratory activity through degradation of the extracellular matrix. Matrix metalloproteinase-2 (MMP-2) and matrix metalloproteinase-9 (MMP-9) have now been shown to regulate tumor cell migration and invasion in other types of cancer [15, 25]. Next, we evaluated the effect of eriodictyol on RB cell migration and invasion by transwell migration, transwell invasion, and western blot assays. The results showed that, with increasing concentrations of eriodictyol, cell migration and invasion were significantly reduced, and the expression levels of MMP-2 and MMP-9 proteins in the cells were significantly decreased. These findings suggest that eriodictyol reduces the ability of RB cells to invade and migrate.

Apoptosis is an autonomous programmed cell death that maintains the stability of the internal environment controlled by genes, and it is associated with a variety of diseases such as tumors and autoimmune diseases [26]. In general, induction of apoptosis in tumor cells is a key mechanism for many targeted drugs against cancer. Finally, we evaluated the effect of eriodictyol on RB cell apoptosis by detecting the expression level of caspase-3 protein. Our results suggest that eriodictyol induces apoptosis in retinoblastoma cells by promoting the shear activation of caspase-3 protein.

In summary, the anticancer effect that eriodictyol can exert on RB cells is the result of eriodictyol's ability to inhibit the proliferation, migration, and invasion of RB cells and induce apoptosis.

PI3K is a phosphatidylinositol kinase that phosphorylates the third hydroxyl group of the inositol ring and has not only phosphatidylinositol kinase activity but also serine/threonine kinase activity. PI3K activates Akt by phosphorylating the serine and threonine phosphorylation sites of Akt in concert with 3-PDK1 [15, 25]. Activated Akt enters the nucleus and activates or inhibits downstream caspases, mTOR, AMPK, and many other proteins involved in cell proliferation, survival, and metabolism [17, 27–29]. Current studies have shown that the expression of the PI3K/Akt signaling pathway-related proteins is abnormally upregulated in a variety of cancers and that activation of the PI3K signaling pathway promotes cancer cell proliferation and inhibits cancer cell death [30, 31]. Therefore, targeted inhibition of PI3K/Akt signaling pathway activation may be a promising strategy for the treatment of cancer [32]. In the next study, we explored the effect of eriodictyol on the PI3K/Akt signaling pathway in RB cells, and we examined the expression levels of PI3K, P-PI3K, Akt, and P-Akt proteins in RB cells to assess whether eriodictyol could inhibit the activation of the PI3K/Akt signaling pathway. The results showed that eriodictyol decreased P-PI3K and P-Akt protein expression levels in a dose-dependent manner, while PI3K and Akt protein expression levels were not significantly changed. These results suggest that eriodictyol can inhibit the activation of the PI3K/Akt pathway in RB cells by inhibiting the phosphorylation of PI3K and Akt.

The article "Effect of Eriodictyol on Retinoblastoma via the PI3K/Akt Pathway" was retracted in 2023. Reasons: signs of a paper mill; suspected computer-generated content; unreliable results or conclusions; lack of ethics approval or compliance.

Zhang et al. showed that eriodictyol exerts anticancer activity against the A549 human lung cancer cell line by inhibiting the activation of the m-TOR/PI3K/Akt signaling pathway [14]. Therefore, we hypothesized that the mechanism of the anticancer effect of eriodictyol on RB cells might be mediated by the PI3K/Akt signaling pathway. Subsequently, we evaluated whether eriodictyol exerts anticancer effects in retinoblastoma by inhibiting the activation of the PI3K/Akt signaling pathway.

Based on the above findings, we found that 100 *μ*M of eriodictyol inhibited the phosphorylation of PI3K and Akt, inhibiting the activation of the PI3K/Akt pathway in RB cells, inhibiting the proliferation, migration, and invasion of RB cells, and inducing apoptosis as a result of the optimal concentration. Therefore, in the next study, we used 100 *μ*M of eriodictyol for the mechanism. The results showed that eriodictyol inhibited the proliferation, migration, and invasion of RB cells and induced apoptosis, probably by inhibiting the phosphorylation of PI3K and Akt proteins. This is consistent with the result that eriodictyol inhibits proliferation and metastasis and induces apoptosis in glioma cells through the PI3K/Akt/NF-*κ*B signaling pathway [9]. In parallel, we used the PI3K agonist 740 Y-P to reverse validate the anticancer effects exerted by eriodictyol in relation to the PI3K/Akt signaling pathway. Interestingly, the combination of eriodictyol and PI3K activator 740 Y-P significantly elevated the protein expression levels of P-PI3K and P-Akt, partially reversed the eriodictyol-induced decrease in proliferation, migration, and invasion of RB cells, and inhibited eriodictyol-induced apoptosis compared to the single administration group. The agonist 740 Y-P targeted increased the phosphorylation of PI3K and decreased the potency of eriodictyol, which fully validated that eriodictyol could exert its anticancer effects on retinoblastoma by inhibiting the PI3K/Akt signaling pathway.

The article "Effect of Eriodictyol on Retinoblastoma via the PI3K/Akt Pathway" was retracted in 2023. Reasons: signs of a paper mill; suspected computer-generated content; unreliable results or conclusions; lack of ethics approval or compliance.

In conclusion, our study shows that eriodictyol inhibits proliferation, migration, invasion, and induction of apoptosis in retinoblastoma through regulation of the PI3K/Akt pathway. However, this study was only explored at the in vitro cellular level, and in the following studies, we will perform further studies in animals to provide a stronger theoretical basis for the anticancer activity of eriodictyol against RB.

## 4. Conclusion

Eriodictyol inhibits proliferation, migration, invasion, and induction of apoptosis in retinoblastoma through regulation of the PI3K/Akt pathway.

## Figures and Tables

**Figure 1:** (a) CCK-8 detection of the effect of eriodictyol on the survival rate of retinoblastoma cells. “^*∗*^” indicates the difference compared with the control group (*P* < 0.05). (b) Western blot detection of the effect of eriodictyol on PCNA protein expression in retinoblastoma cells. “^*∗*^” indicates the difference compared with the control group (*P* < 0.05).

**Figure 2:** Transwell migration assay of the effect of eriodictyol on retinoblastoma cell migration; the scale bar of the migration-invasion map is 100 *μ*M with 200-fold magnification.

**Figure 3:** (a) Western blot detection of the effect of eriodictyol on MMP-2 and MMP-9 protein expression in retinoblastoma cells. “^*∗*^” indicates the difference compared to the control (*P* < 0.05). (b) Transwell invasion assay of the effect of eriodictyol on retinoblastoma cell invasion. “^*∗*^” indicates a difference compared with the control group (*P* < 0.05). The scale bar of the migration-invasion map is 100 *μ*M with 200-fold magnification.

**Figure 4:** (a) Flow cytometry detection of the effect of eriodictyol on apoptosis of retinoblastoma cells. (b) Quantification of flow cytometry results. (c) Western blot detection of the effect of eriodictyol on cleaved caspase-3 protein expression in retinoblastoma cells. “^*∗*^” indicates a difference compared with the control group (*P* < 0.05).

**Figure 5:** (a) Western blot detection of the effect of eriodictyol on P-PI3K, PI3K, P-Akt, and Akt protein expression in retinoblastoma cells. (b) Western blot detection of the effect of eriodictyol on P-PI3K/PI3K and P-Akt/Akt protein expression ratio in retinoblastoma cells. “^*∗*^” indicates a difference compared to the control group (*P* < 0.05).

**Figure 6:** (a) Western blot detection of the effect of PI3K agonist 740 Y-P in combination with eriodictyol on PI3K and Akt protein expression in retinoblastoma cells. (b) CCK-8 detection of the effect of PI3K agonist 740 Y-P in combination with eriodictyol on the survival rate of retinoblastoma cells. (c) Transwell migration to detect the effects of PI3K agonist 740 Y-P in combination with eriodictyol on retinoblastoma cell migration and invasion, respectively. (d) Transwell invasion to detect the effects of PI3K agonist 740 Y-P in combination with eriodictyol on retinoblastoma cell migration and invasion, respectively. (e) Flow cytometry to detect the effects of PI3K agonist 740 Y-P in combination with eriodictyol on apoptosis of retinoblastoma cells; “^*∗*^” indicates a difference compared with the control or 100 *μ*M eriodictyol group (*P* < 0.05).

The article "Effect of Eriodictyol on Retinoblastoma via the PI3K/Akt Pathway" was retracted in 2023. Reasons: signs of a paper mill; suspected computer-generated content; unreliable results or conclusions; lack of ethics approval or compliance.

## Data Availability

The simulation experiment data used to support the findings of this study are available from the corresponding author upon request.
